# Prediction of Retail Price of Sporting Goods Based on LSTM Network

**DOI:** 10.1155/2022/4298235

**Published:** 2022-07-09

**Authors:** Hui Ding

**Affiliations:** School of Physical Education, Henan University of Science and Technology, Luoyang, Henan 471000, China

## Abstract

Commodity prices play a unique role as a lever to regulate the economy. Price forecasting is an important part of macrodecision-making and micromanagement. Because there are many factors affecting the price of goods, price prediction has become a difficulty in research. According to the characteristics that price data are also affected by other factors except for time series, a multifactor LSTM price prediction method is proposed based on the long-term and short-term memory network (LSTM) deep learning algorithm. This method not only makes use of the memory of LSTM to historical data but also introduces the influence of external factors on price through the full connection layer, which provides a new idea for solving the problem of price prediction. Compared with BP neural network, the experimental results show that this method has higher accuracy and better stability. Analyze the commodity description and commodity price characteristics, find out the commodities similar to the target commodity, complete the commodity price data by using the historical price data of similar commodities, and establish the training set to verify the validity of the proposed method.

## 1. Introduction

The market scale of the commodity market is expanding day by day, the trading varieties are becoming richer and richer, and the trading mechanism is becoming more and more standardized. Since the development of the commodity market, it has become an important financial submarket. The price signal spread in the market plays an important guiding role in guiding enterprise production, international trade, and regulating the economy [1]. China's commodity exchanges have also accumulated rich market data in many years of operation and development. Researchers collect, sort out, and analyze the transaction data of various commodities and then add and compile the same commodity indexes. These indexes can reflect the overall state of relevant commodity price fluctuations and the development trend of the commodity economy and help government functional institutions understand the tail state of the macroeconomy; at the same time, relevant enterprises can also use the rice commodity price information contained in the commodity index to make their own business decisions, reasonably arrange the purchased quantity and minimize unnecessary economic losses [2, 3].

Commercial activities occupy a more and more important position in the national economy. Commercial behavior not only makes an important contribution to the national economy in terms of output but also plays an important role in breeding market relations, improving market mechanism, and solving the problem of labor employment [4]. Today, with the high development of information technology, e-retail commerce, as a new retail commodity sales model, has developed rapidly. People can obtain thousands of commodity information through the Internet and contact commodity sellers all over the world for transactions without going out of their homes [5]. The emergence of e-commerce has greatly facilitated the people's life, promoted people's consumption enthusiasm, and increased the vitality of the consumer market; the development of e-retail commerce has driven the prosperity of the business market. Tens of thousands of retail commodities are displayed and sold on the Internet, which reduces the cost of commodity sales and improves the efficiency of sales. At the same time, because e-retail commerce relies on the Internet, it has natural advantages in the acquisition and storage of information and data. Enterprises obtain a large amount of data through information technology. How to mine these data and find valuable laws, so as to guide the business decision-making of enterprises, improve the sales model, formulate effective sales strategies, and finally obtain economic benefits from e-commerce. Many enterprises begin to invest in the direction of commercial data mining and develop their own commercial data mining schemes.

Exploratory data analysis is an important stage of data analysis, which is different from initial data analysis. The focus of preliminary data analysis is on whether the requirements for identifying statistical models and hypotheses are met to ensure the reliability of confirmatory analysis [6–8]. In this analysis process, the unqualified data are filled with missing value, data conversion, outlier value discarding, and other processing to enhance the accuracy of the analysis. Exploratory data analysis includes preliminary data analysis, but its starting point is not only to determine data quality but also to discover patterns of data distribution (Patten) and propose new hypotheses from the data. Exploratory data analysis is identified as a key step in the data science workflow that can affect multiple processes. In the data science workflow shown in Figure 1, exploratory data analysis is closely related to other processes.

Each base model trains the input variables of the training set separately. Through supervised learning, each base model. A weight is established for the predicted value of the training set of each base model by means of a weighted average, and then the established weight value is assigned to the predicted value of the test set of each base model [9, 10]. Forecast weight value multiplication and intercept Get model test set of predicted values.  Figure 2 shows the construction flow and diagram of the model. From the figure we know that it mainly includes the data preprocessing, the multiple prediction results from multiple LSTM models and the prediction results are integrated and enhanced by weighting multiple parameters.

By analyzing the weight value of each base model of sports products, it is found that the base model with higher prediction accuracy is more likely to get more weight.  Figure 3 is the technology roadmap.

## 2. Related Work

Price prediction refers to the prediction behavior of dynamic analysis of future price changes according to the historical value and price trend of commodities [11]. The authors of [12] used the recurrent neural network model for high-speed train vibration prediction from time series and achieved good results.

With the development of a simple time series algorithm, the application of simple time series analysis is gradually expanding. At present simple time series analysis algorithm has been in agricultural prices, industrial commodity prices prediction, financial stock price forecasting, and many other fields have a wide range of applications, due to less used in the analysis of data information, at the same time the low effective information analysis to history, lead to predicting the results still cannot meet the needs of social development.

Research status of price forecasting algorithm based on simple time series: according to the periodicity and seasonality of power price fluctuation, Marcjasz et al. [13, 14] analyzed the influence of seasonality on future power price change and used NARX neural networks model to predict power price, which achieved good results. In order to obtain good prediction result, the authors of [15] designed a Denoising Aggregation of Graph neural networks by using the principal component analysis. Wang et al. [16–18] studied the short-term electricity price forecasting with stacked denoising autoencoders, do the research and application of a hybrid forecasting framework, and proposed the novel hybrid model for air quality index two-phase decomposition technique and modified extreme learning machine (ELM), respectively. Chong et al. [19, 20] studied the deep learning networks for stock market analysis and prediction and carried the empirical asset pricing via machine learning, respectively. Nilashi et al. presented an analytical approach for big social data analysis for customer decision-making in eco-friendly hotels and tested the proposed solution on two open datasets [21]. In addition to the above works, Hoseinzade [22] combined the ANN model and CNN model, predicted the rise and fall of Shanghai Futures in the known period and achieved good prediction results. Investors can also make investment decisions with the help of Chen and Ge [23] explored the attention mechanism in LSTM-based Hong Kong stock price movement prediction. Fang et al. do the research on quantitative investment strategies based on deep learning [24]. Based on the above-given discussions, the main contributions of this paper are summarized as follows:

1. As an improved structure of the RNN model, the LSTM model not only inherits the characteristics of the RNN model suitable for dealing with time series data but also further solves the problem of a long-term dependence on time dimension and improves the accuracy of prediction. Its prediction effect is superior to BP neural network, RNN, CNN, GRU, and other neural network models.
2. Grid Search is used to train the model with different parameters and cross-validating each model until the optimal combination of values is found to ensure the best model performance.
3. The optimized model is verified on the test set, and the mean square error is used as the evaluation index to prevent the model from overfitting. The results show that the model achieves low mean square error in both the training set and the test set, and obtains ideal prediction results.

## 3. LSTM Network

LSTM neural network was first proposed by Hochreiter et al. (1997) and further extended after its optimization and improvement by Alex graves. In many practical problems related to sequence data, LSTM has achieved great success and has been widely used, such as natural language processing (NLP), time series prediction, and so on.

The traditional recurrent neural network (RNN) can not deal with the long-term sequence problem, to solve this problem, the LSTM neural network is proposed by adding a “gate” structure to control the cell state and output at different times to alleviate the problem of gradient disappearance. The “gate” structure of LSTM includes three types: “forgetting gate,” “input gate,” and “output gate.” The function of the “forgetting gate” is to judge the information transmitted from the previous time to the current time and selectively “forget” some information is shown in Figure 4. In addition, the orthogonal initialization is proposed to avoid gradient disappearance or explosion at the initial stage of training, ReLU (Rectified Linear Unit) activation function can alleviate gradient disappearance, gradient shear can solve gradient explosion, and the LSTM Unit can control gradient disappearance. LSTM has been successfully applied in machine translation, conversation generation, and other fields, showing excellent modeling ability of sequence data. Therefore, this paper builds a retail price of a sporting goods prediction model based on the LSTM network unit and can make full use of its feature that any length sequence can be used as input and apply it to online data recognition. LSTM solves the problem that RNN cannot handle long time dependence by introducing [25].

Let the number of input neurons in the whole hidden layer be *G*, *G* includes all units and gates and use index *G* to represent these input neurons. The forward calculation of LSTM is to calculate an input sequence *X* with a length of time *d*, whose starting point is *t* = 1 [26, 27]. When the value of time point *T* increases continuously, the equation will be updated recursively until *t* = *t*. Like forward calculation, reverse calculation is an input sequence *X* with a time length of *T*, but the starting point of reverse calculation is *T* = *T*. When the value of *T* decreases continuously, the reciprocal of the unit is calculated recursively until *T* = 1. According to the derivatives at each time point above, we can obtain the final weight derivative value.

(1) $$\begin{array}{c} \delta_{j}^{t}≜\frac{\partial l}{\partial a_{j}^{t}}, \end{array}$$

where *l* is the loss function used for training.

The value of the input gate at time *t* is

(2) $$\begin{array}{c} i_{t}=\sigma \left(W_{i}\times \left(h_{t-1},X_{t}\right)+b_{i}\right),\\ a_{t}=\tanh\left(W_{c}\times \left(h_{t-1},X_{t}\right)+b_{c}\right). \end{array}$$

### 3.1. Forgetting Gate

The forgetting gate controls what information is left out and calculate the activation value *f* of the forgetting gate at time *t*.

(3) $$\begin{array}{c} f_{t}=\sigma \left(W_{f}\times \left(h_{t-1},X_{t}\right)+b_{f}\right), \end{array}$$

where *W*_*f*_ and *b*_*f*_ represent the weight and bias of the forgetting gate, respectively, while *σ* represents the Sigmoid function.

### 3.2. Cell State Update

The cell state is updated according to the calculation results of the input gate and forgetting gate, so as to obtain the cell state update value at the moment [28].

(4) $$\begin{array}{c} C_{t}=i_{t}\times a_{t}+f_{t}\times C_{t-1}. \end{array}$$

### 3.3. Output Gate

Control determines which information needs to be output. According to the computed cell status update value *C*_*t*_, the following calculation formula of the output gate can be obtained:

(5) $$\begin{array}{c} h_{t}=\sigma \left(W_{0}\times \left(h_{t-1},X_{t}\right)+b_{0}\right)\tanh\left(C_{t}\right). \end{array}$$

Sigmoid activation function and TANH activation function are used in the gated structure of the neural unit structure of the LSTM neural network. Here, the Sigmoid function is

(6) $$\begin{array}{c} f\left(x\right)=\frac{1}{1+e^{-x}}. \end{array}$$

tanh function is

(7) $$\begin{array}{c} f\left(x\right)=\frac{e^{x}-e^{-x}}{e^{x}+e^{-x}}. \end{array}$$

Before the data are input into the neural network model, the data need to be normalized. Normalization of the features of a numeric type can unify all the features into a roughly identical numeric interval. The normalization of data can eliminate dimensionality, thus avoiding the dependence of data on the choice of units of measurement and help to improve the performance of the model [29].

(8) $$\begin{array}{c} x_{i}^{\prime }=\frac{x_{i}-\bar{x}}{\max\left(x\right)-\min\left(x\right)}, \end{array}$$

where *x*_*i*_ is the *I* variable; *x* is mean of *x*_*i*_; max (*x*) and min (z) represent the maximum and minimum values *x*_*i*_.

By using different neural network models to train the model on the training set and test the model on the test set, the model performance of different neural network models under different parameter settings is compared. In this paper, MAE, MSE, MAPE, and the correlation coefficient (*P*) between predicted data and real data were selected as the evaluation indexes of model performance.

The MAE is

(9) $$\begin{array}{c} e_{\text{MAE}}=\frac{1}{n}\left|y_{i}-{\hat{y}}_{i}\right|. \end{array}$$

The MSE is

(10) $$\begin{array}{c} e_{\text{MSE}}=\frac{1}{n}\sum_{i=1}^{n}{\left(y_{i}-{\hat{y}}_{i}\right)}^{2}. \end{array}$$

The MSPE is

(11) $$\begin{array}{c} e_{\text{MAPE}}=\frac{1}{n}\sum_{i=1}^{n}\left|\frac{y_{i}-{\hat{y}}_{i}}{y_{i}}\right|. \end{array}$$

The correlation coefficient is

(12) $$\begin{array}{c} P=\frac{\text{COV}\left(Y,\hat{Y}\right)}{\sqrt{\text{VAR}\left(Y\right)\cdot \text{VAR}\left(\hat{Y}\right)}}, \end{array}$$

where *n* is the number of test data sets; *y*_*i*_ is the true value of the *i* sample point; ${\hat{y}}_{i}$ the model predicted value of the sample point; **Y** is the true value of sample; $\hat{Y}$ is the predicted value of the model; $\text{COV}\left(Y,\hat{Y}\right)$ is the covariance between *y* and *y*; VAR(**Y**) is the variance of *l*; $\text{VAR}\left(\hat{Y}\right)$ of *y* is the variance of $\hat{Y}$.

## 4. Data Processing and Exploration

The main innovation point of this paper is to improve the conventional LSTM model and apply it to forecast the retail price of sports products, so we mainly compare it with the conventional LSTM model. Secondly, because real data sets are precious and difficult to obtain, this paper uses only one data set for the simulation experiment. Because the quality of the data affects the training of the selected model, the collection, analysis, and processing of the data are the key stages before the model training. The data in this paper mainly include two parts: the research object and the characteristic data [30].

General forecast commodity price focuses on sports commodity price. Use Python to conduct descriptive statistical analysis of different sports commodities and draw their closing price charts [31, 32], as shown in Figure 5. The distribution is skewed to the right, the peakness is smaller than 3, the tail shape is thin, and does not obey the normal distribution.

### 4.1. Data Noise Reduction

As the market dynamics are very complex, these data contain infrequent noises, so the library in Python is used for wavelet transformation to remove data noises [33]. It is worth noting that the conventional wavelet change model is used in this paper. It inherits and develops the idea of short-time Fourier transform localization and overcomes the shortcomings of window size not changing with frequency. It can provide a “time-frequency” window changing with frequency, which is an ideal tool for time-frequency analysis and processing of signals. Therefore, it is especially suitable for removing noise in financial data. Figures 6 and 7 are the comparisons before and after wavelet transformation.

After the LSTM neural network training is completed, the prediction results and corresponding MSE values of model 1 and Model 2 are given, respectively, as shown in Figure 8, and the prediction results of model 1 and Model 2 are shown in Figure 9.

The basic idea of model training is to fit a set of rules system on the training data set to reveal the rules in the data. In other words, the fit describes how well, or how well, the model can be generalized to the data in the test set. A good model results in good model performance and can be validated with new data outside the training data set, i.e., out-of-sample data. In addition to parameters that can be learned, different models require different hyperparameters, which are parameters that do not need to be trained. Parameters are critical to the model and depend on training data. As part of the training process, the LSTM model is further adjusted and optimized to obtain a better prediction effect by learning parameters from training data through optimization techniques [34–37].

The process of economic research is generally to explain economic phenomena by constructing economic models. When generally accepted economic phenomena are confirmed by scholars, they need to be listed in the form of typical facts. In the followup research, if the solution of the model in the general equilibrium state is consistent with the typical facts, it can explain that the model is more reasonable to a great extent. In the study of financial problems, especially in the study of financial time return series, some common statistical characteristics can often be observed. According to scholars' typical facts of univariate return series, they are summarized as follows: they often show autocorrelation; It often shows long memory; The slow decay of absolute return autocorrelation; peak thick tail distribution; the distribution shape changes with time; wave aggregation effect; after adjusting the fluctuation aggregation, there is still a conditional thick tail effect. Under the assumption of independent and identically distributed, the performance of the fitted financial time series model is often not optimal, so the distribution characteristics of the data need to be considered when modeling the income series. When the neural network model is used to model the data, the assumption of distribution does not need to be considered. This is because the neural network model has the ability to generalize the structure of input data so that the nonlinear characteristics of financial data can be captured by the neural network.

Grid Search is a method of systematically training a model, using different combinations of hyperparameter values to train the model, cross-validating each model until the optimal combination of values is found to ensure the best model performance. Can through continuous testing parameters of all combinations, a group to find the most appropriate combination of super configuration parameters will be discretization, super parameters according to their own characteristics to select several experience values, and then according to different combinations of the training model, so as to select an optimal combination of configuration, the circumstances of less suitable for super parameters. Random Search is to randomly combine hyperparameters and then select the optimal configuration. It does not make unnecessary attempts on unimportant parameters because, just as regularization coefficients have a limited impact on model performance, learning rates have a greater impact on model performance, so it does not make unnecessary attempts. Random searches are generally more efficient and easier to implement than grid searches. However, these two methods do not consider whether there is a correlation between hyperparameters, so they are relatively inefficient. Bayesian optimization is an adaptive hyperparameter optimization method, which predicts the next possible hyperparameter combination based on the tested hyperparameter combination in order to obtain the maximum utility. Since the cumulative distribution function of Gaussian distribution is an s-type function, the GELU function can be approximated by tanh function or Logistic function as shown in Figure 10.

The simplest strategy is to fix a learning rate throughout the training process. Choosing a smaller learning rate allows the optimizer to find a good solution, but it is easy to limit the convergence rate. The relationship between the two can be balanced by taking time to change the learning rate.  Figure 11 shows the learning rate for each period.

After many times of adjustment and optimization, the prediction results before and after improvement are shown in Figures 12 and 13, respectively. The final model structure and parameters obtained are as follows: the Sequential length of the test window is 55, and the sequential model consists of three LSTM layers, with the number of neurons in each layer being 100, 100, and 150, respectively. In order to avoid overfitting, two Dropout layers are added with the Dropout layer of 0.2, and the dimension of input data are 5. The dense layer was added to aggregate its dimension into 1, the activation function was linear, and the loss function was set as Mean Squared Error (MSE). Adam was used as the optimization algorithm, and two Epochs were used as the model. Each batch is 32 in size.

The conventional price forecasting model is also a deep learning model. Firstly, a conventional price prediction model is constructed; that is, the model only contains market data and financial data. The previous market data and financial data are used to train the deep learning model to get the trained deep learning model to predict the future market; Through natural language processing technology, emotional information extraction and emotional evaluation are carried out on public opinion data. Combined with the conventional price prediction model, the in-depth learning model is trained by using market data, financial data, research reports, and emotional tendency data of financial news, and the model is used to predict the future market. Then, the prediction effect of the conventional securities price prediction model is compared with that of the deep learning model based on the natural language processing results of public opinion data.

After determining the number of input nodes, output nodes, and hidden layer nodes of the two models LSTM network, the deep learning model can be trained. After many experiments, it is found that the training times are too few and the model training error is too large, so it is necessary to continuously increase the training times, but with the increase of the training times; the error of model training gradually tends to a stable value. If the training times of the model are increased a lot at this time, the model effect is not improved much. It is the result of training the first model of CCCC. When the training times are less than 200, the error of the model is large. At this time, increasing the training times will quickly reduce the error of model training; When the training times are more than 200 times and less than 1000 times, the model error has been small. At this time, when the training times are increased, the reduction degree of model training error has shown a decreasing law; When training 1000 to 2000 times, the error of the model changes in a small area, and the effect of increasing the number of training times are gradually not obvious. Through many tests and comparisons, it is found that when the number of training times of the model is about 2000 times, it can meet the accuracy requirements of training. If the number of training times is increased, the effect of improving the model training error is small, Moreover, it takes a long time to train the model in the computer, so it is of little significance to increase too many training times. Therefore, we set the training times of the in-depth learning model in this study at 2000 times. In the later model, we also verify that it conforms to this law. Therefore, the second in-depth learning model with public opinion information data also set the training times at 2000 times.

## 5. Conclusion

1. This paper applies deep learning theory, based on the characteristics of financial time series data, uses LSTM neural network model to predict sports commodity price index, and compares its prediction results with the prediction results using the network model. Experimental results show that LSTM neural network model has the best performance on the test set.
2. A prediction model is established. On the basis of collated data feature engineering, a neural network prediction model based on long and short-term memory is established, and the model is trained with a training set to predict the price of sports goods. In terms of model optimization, the number of hidden layer neurons, learning rate, batch size, and training wheel were adjusted to achieve the best training results.
3. In this sports commodity price trend prediction model, different sports price data will have different influences on the prediction effect, so the selection of the data set is also very important.

Although the model proposed in this paper achieves good prediction results, the model does not consider the correlation of data time. Some sliding time window tools can be used in future studies to improve the prediction step size and prediction accuracy of the model.

## Figures and Tables

**Figure 1:** Data science workflow.

**Figure 2:** Flow chart of model construction.

**Figure 3:** Empirical technology Roadmap.

**Figure 4:** LSTM structure diagram.

**Figure 5:** Price trend.

**Figure 6:** Wavelet transforms before.

**Figure 7:** Wavelet transforms after three-layer decomposition.

**Figure 8:** Fitting diagram of Model 1 and Model 2 training sets.

**Figure 9:** Prediction results of Model I and Model II.

**Figure 10:** ReLU function and GELU function.

**Figure 11:** Learning rate.

**Figure 12:** Prediction results before model improvement.

**Figure 13:** Prediction results after model improvement.

## Data Availability

The data used to support the findings of this study are available from the author upon request.
